The article "Comparison of Image Quality and Radiation Dose Between Single-Energy and Dual-Energy Images for the Brain With Stereotactic Frames on Dual-Energy Cerebral CT" was published in 2022. Journal: Front Radiol.

# Comparison of Image Quality and Radiation Dose Between Single-Energy and Dual-Energy Images for the Brain With Stereotactic Frames on Dual-Energy Cerebral CT

**DOI:** 10.3389/fradi.2022.899100

**Published:** 2022-06-10

**Authors:** Xiaojing Zhao, Wang Chao, Yi Shan, Jingkai Li, Cheng Zhao, Miao Zhang, Jie Lu

**Affiliations:** ^1^Department of Radiology & Nuclear Medicine, XuanWu Hospital of Capital Medical University, Beijing, China; ^2^Beijing Key Laboratory of Magnetic Resonance Imaging and Brain Informatics, Beijing, China

**Keywords:** radiography, dual-energy scanned projection, artifacts, neuronavigation, imaging enhancement

## Abstract

**Background:**

Preoperative stereotactic planning of deep brain stimulation (DBS) using computed tomography (CT) imaging in patients with Parkinson's disease (PD) is of clinical interest. However, frame-induced metal artifacts are common in clinical practice, which can be challenging for neurosurgeons to visualize brain structures.

**Objectives:**

To evaluate the image quality and radiation exposure of patients with stereotactic frame brain CT acquired using a dual-source CT (DSCT) system in single- and dual-energy modes.

**Materials and Methods:**

We included 60 consecutive patients with Parkinson's disease (PD) and randomized them into two groups. CT images of the brain were performed using DSCT (Group A, an 80/Sn150 kVp dual-energy mode; Group B, a 120 kVp single-energy mode). One set of single-energy images (120 kVp) and 10 sets of virtual monochromatic images (50–140 keV) were obtained. Subjective image analysis of overall image quality was performed using a five-point Likert scale. For objective image quality evaluation, CT values, image noise, signal-to-noise ratio (SNR), and contrast-to-noise (CNR) were calculated. The radiation dose was recorded for each patient.

**Results:**

The mean effective radiation dose was reduced in the dual-energy mode (1.73 mSv ± 0.45 mSv) compared to the single-energy mode (3.16 mSv ± 0.64 mSv) (*p* < 0.001). Image noise was reduced by 46–52% for 120–140 keV VMI compared to 120 kVp images (both *p* < 0.01). CT values were higher at 100–140 keV than at 120 kVp images. At 120–140 keV, CT values of brain tissue showed significant differences at the level of the most severe metal artifacts (all *p* < 0.05). SNR was also higher in the dual-energy mode 90–140 keV compared to 120 kVp images, showing a significant difference between the two groups at 120–140 keV (all *p* < 0.01). The CNR was significantly better in Group A for 60–140 keV VMI compared to Group B (both *p* < 0.001). The highest subjective image scores were found in the 120 keV images, while 110–140 keV images had significantly higher scores than 120 kVp images (all *p* < 0.05).

**Conclusion:**

DSCT images using dual-energy modes provide better objective and subjective image quality for patients with PD at lower radiation doses compared to single-energy modes and facilitate brain tissue visualization with stereotactic frame DBS procedures.

## Introduction

Parkinson's disease (PD) is a progressive nervous system disorder that affects more than 53 million people, which has resulted in about 103,000 deaths globally in 2013. Moreover, in China, the number of patients with PD will reach 4.94 million in 2030. For patients with advanced PD, deep brain stimulation (DBS) was a standard surgical treatment, especially when drug therapy failed to provide sufficient benefits. During the surgery, electrodes would be inserted into the specific part of the brain with the help of a stereotactic head frame, for instance, the subthalamic nucleus, which is the preferred stimulation target for patients with PD in the late stage (1, 2).

Typically, patients would undergo magnetic resonance imaging (MRI) under frameless conditions to provide a detailed deep brain anatomy, particularly the anterior and posterior cerebral convergence, the pallidum and the third ventricle. Then, non-enhanced brain CT scans were performed together with the stereotactic head frames. Finally, fused CT and MRI images were used to localize the subthalamic nuclei and guide the neuronavigation system as a standard technique (3). However, distortion of MRI images caused by high magnetic field strength may mislead to failure of preoperative image fusion. In this case, the quality of CT images becomes particularly important.

Although conventional CT is significant, it has also some problems such as metal artifacts. X-ray photons lose a significant amount of energy after penetrating metal materials, creating a combination of beam hardening and photon starvation effects. This leads to severe dark or bright streak artifacts behind the stainless steel pegs holding the head frame in place, which affects the display of intracranial brain tissue (4, 5). Using single-energy CT (SECT), attempts have been made to reduce metal artifacts by increasing the tube current or tube voltage peak. However, the improvement in image quality was not significant and came at the cost of increased radiation dose. Another useful attempt to improve the image quality of preoperative navigation is dual-energy CT (DECT). Unlike SECT, DECT is a promising imaging technique that simultaneously images patients using two different X-ray energies (6) and reconstructs virtual monoenergetic images (VMI) at 40–190 keV by exploiting the difference in attenuation of the material at high and low energies. High-virtual high-kiloelectron voltage (keV) monoenergetic images have been shown to be effective in reducing artifacts of metallic implants (6, 7). Several studies have demonstrated that evidence of VMI reconstruction has the potential to eliminate metal artifacts in some small-sized implants in the head, such as implanted teeth and platinum coils or clips (8–10). However, few studies have discussed the value of the dual-energy mode in eliminating severe metal streak artifacts caused by stereotactic head frames and comparing radiation dose and image quality with the single-energy mode.

Therefore, the aim of our study was to evaluate the radiation dose and image quality of patients with stereotactic head frames obtained using the DSCT system in single- and dual-energy modes.

## Materials and Methods

### Patient Population

Totally, 60 patients with consecutive PD (29 males, 31 females) were included between March 2018 and April 2019 in this study and randomly separated into two groups. Thirty patients (39 to 72 years old) who took the dual-energy mode (80/Sn150 kVp) of head CT and another 30 patients (33 to 78 years old) who took head CT images under 120 kVp were included; all the patients were planned to take surgical treatment in functional neurosurgery. All of the patients underwent CT navigation scanning before performing the stereotactic guided DBS surgery. This study was approved by the Ethics Committee of our hospital, and informed consent was given to all the patients prior to inclusion into the study.

### CT Scan Protocols and Reconstruction

All the patients were scanned using the third-generation DECT (SOMATOM Force, Siemens Healthineers) in the non-contrast head CT dual-energy mode. The dual energy mode tube voltage was set to 80 kVp and Sn150 kVp; the use of a tin filter can further harden the beam and increase the mean energy. The tube current was set to CARE Dose4D. Other scan parameters were:collimation, 64 mm × 0.6 mm; pitch, 0.7, rotation time, 0.5 s/r; reconstruction matrix, 512 × 512. Dual-energy images were loaded on the dedicated workstation (Syngo.via, Siemens Healthineers) for post-processing.

The single-energy mode tube voltage was set to 120 kVp; pitch, 0.55, and the tube current was set to CARE Dose4D. All the images were further reconstructed in axial orientation at a slice thickness of 1 mm and an increment of 1 mm.

### Radiation Dose Assessment

The volumetric CT dose index (CTDI vol) and dose length product (DLP) in both groups were recorded from the dose reports of protocols. The effective dose (ED) estimation was calculated by the formula: ED = k × DLP, k = 0.0019 mSv × mGy^−1^ × cm^−1^; k was a head specific conversion coefficient (11).

### Subjective Image Quality Evaluation

The MonoenergeticPlus algorithm (Mono+, Siemens Healthineers) was applied to generate VMIs from 50 keV to 140 keV at 10-keV intervals. Thus, 10 sets of VMIs, together with single-energy CT images (120 kVp), were observed and evaluated by two experienced radiologists at the head window center and width (W:100, L:35). Radiologist A has 8 years of diagnostic experience in brain CT imaging and Radiologist B has 19 years of diagnostic experience in head CT and MRI imaging. Both observers were blinded to the keV level and assessed individually. All the images' subjective evaluation used the following five-point Likert grading (Table 1).

**Table 1:** 5-point Likert grading criteria.

Score 1:	Examination non-diagnostic;
Score 2:	Restricted diagnostic interpretation;
Score 3:	Minor artifacts without affecting neural or vascular structures;
Score 4:	Minor artifacts phantoms to completed diagnostic evaluation;
Score 5:	No artifacts perceivable (10).

### Objective CT Image Analysis

The mean attenuation values, image noises, signal-to-noise ratio (SNR), and contrast to noise (CNR) were served as indices for evaluating image quality and the severity of metal artifacts (10). For all the patients, two observers drew four regions of interest (ROIs) at the severest artifact area close to stereotactic nails, one background ROI on brain tissue away from metal artifacts was selected to get the SNR and CNR, and each ROI was limited to a 1-cm^2^ circle (Figure 1). The location of dual-energy ROIs at different energy levels images (50–140 keV) remains unchanged. The CT values and image noise were recorded; the image noise was represented by the standard deviation (SD) within the ROIs. To minimize the effect of discordant measurement, the final record was the average of four ROIs. The SNR and CNR were calculated using the following formula: $\text{SNR}=\frac{\text{CT values}(\text{ROI})}{\text{SD}(\text{ROI})\;}$, $\text{CNR}=\frac{\text{CT values}(\text{ROI})-\text{CT values}(\text{background})}{\sqrt{\text{SD}{\left(\text{ROI}\right)}^{2}+\;\text{SD}{\left(\text{background}\right)}^{2}}}$(11).

**Figure 1:** Four regions of interest (ROIs) near the stereotactic nail **(A–D)** and one background ROI on brain tissue **(E)** were selected.

### Statistical Analysis

Statistical analysis was performed using commercial software (SPSS20.0 statistical software, USA). Interval variables were expressed as mean ± SD. Inter-observer agreement on image quality and artifact severity was determined by Kappa statistic: *K* ≤ 0.2 means poor agreement; 0.21 < *K* ≤ 0.40 means fair agreement; 0.41 < *K* ≤ 0.60 means moderate agreement; 0.61 < *K* ≤ 0.80 means good agreement; *K* > 0.81 means excellent agreement.

Objective measurements among VMIs were used in the repeated measures ANOVA. Wilcoxon signed-rank test was used on the subjective evaluation to compare the difference of the image score between single-energy images and dual-energy monochromatic images. A Pairwise comparison was carried out to compare the radiation dose between Group A and Group B. A *P* value < 0.05 was considered statistically significant difference.

## Results

### Patients

Table 2 gives an overview of 60 patient characteristics. Difference of gender and patient age between groups did not reach statistical significance (*p* > 0.05).

**Table 2:** Baseline characteristics.

**Characteristic**	**Dual-Energy mode**	**120kVp**	***P-*** **value**
Age(years)	51.96 ± 14.08	60.73 ± 10.46	0.11
Gender	12M |18F	19M | 11F	0.051

### Radiation Dose

The dual-energy mode radiation dose is as follows: the CTDI_vol_ and DLP were (30.19 ± 5.45) mGy and (913.98 ± 235.90) mGy × cm; the ED was (1.73 ± 0.45) mSv. The dual-energy mode (Group A) showed significantly lower radiation exposure compared to the single-energy mode (Group B) (all *p* < 0.001). All radiation dose parameters are summarized in Table 3.

**Table 3:** Radiation dose values.

	**Group A (dual-energy mode)**	**Group B** **(single-energy mode)**	***F***	***Sig***	***P***
CTDI_vol_(mGy)	30.19 ± 5.45	50.68 ± 8.29	2.74	0.10	<0.001
DLP(mGy × cm)	913.98 ± 235.90	1663.19 ± 337.96	2.13	0.15	<0.001
Effective dose (mSv)	1.73 ± 0.45	3.16 ± 0.64	2.13	0.15	<0.001

### Objective Image Quality Evaluation

The results of objective image quality parameters are listed in Table 4. The CT values, SNR, CNR of all the regions increased as keV increased. The CT values of 100–140 keV were higher than that of 120 kVp images. At 90–100 keV, there was no significant difference in CT values, but, at 120–140 keV, showed a significant difference (all *p* ≤ 0.02). The SNR was higher at 90–140 keV of the dual-energy mode compared with 120 kVp images. At 90–100 keV, there was no significant difference in SNR, but showed significant differences among the two groups at 120–140 keV (all *p* ≤ 0.01). The CNR of 60–140 keV VMIs was significantly better in the Group A compared to Group B (all *p* < 0.001). The image noise of all the regions decreased as keV increased. The image noise of 90–140 keV was lower than that of 120 kVp images, and, at 100–140 keV, did reach statistical significance (all *p* < 0.01).

**Table 4:** Objective image quality parameters.

**Energy level**	**CT values**	**Image noise**	**SNR**	**CNR**
120 kVp	−74.37 ± 81.92	47.58 ± 40.62	−1.58 ± 1.63	−3.40 ± 1.74
50 keV	−403.89 ± 277.59^a^	113.57 ± 64.65^a^	−3.31 ± 2.10^a^	−2.76 ± 1.86
60 keV	−272.05 ± 185.28^a^	81.16 ± 47.33^a^	−3.03 ± 1.99^a^	−2.39 ± 1.64^a^
70 keV	−185.37 ± 141.58^a^	61.44 ± 37.80^a^	−2.63 ± 2.14^a^	−1.97 ± 1.62^a^
80 keV	−131.26 ± 102.67^a^	49.58 ± 31.52	−2.12 ± 2.16	−1.54 ± 1.42^a^
90 keV	−86.12 ± 77.25	40.80 ± 26.96	−1.47 ± 2.33	−1.10 ± 1.27^a^
100 keV	−52.06 ± 58.80	32.66 ± 23.70^a^	−0.78 ± 2.62	−0.70 ± 1.22^a^
110 keV	−29.52 ± 47.74	28.18 ± 22.08^a^	−0.02 ± 2.81^a^	−0.35 ± 1.20^a^
120 keV	−13.41 ± 39.84^a^	25.35 ± 20.73^a^	0.63 ± 2.80^a^	−0.06 ± 1.18^a^
130 keV	−1.72 ± 34.70^a^	23.62 ± 19.68^a^	1.17 ± 2.81^a^	0.17 ± 1.18^a^
140 keV	7.29 ± 30.81^a^	22.69 ± 18.77^a^	1.53 ± 2.61^a^	0.35 ± 1.18^a^

a *Represented that the objective evaluation at this keV was statistically significant compared with 120 kVp images (p < 0.05)*.

### Subjective Image Quality Evaluation

The dual-energy mode that generated 50–140 keV VMI subjective evaluation was included in our study. As shown in Figure 2, the metal beam-hardening artifacts were mainly located at the long-axis direction of stainless nails. The 120 kVp images and 50–80 keV monoenergetic images had the severest streak artifacts, which decreased the image quality. Table 5 shows that the subjective scores gradually increased as virtual monochromatic energy increased. The highest subjective scores were at 120 keV, and, at 110–140 keV, were significantly higher than the images at the polychromatic 120 kVp CT images (all *p* < 0.05). The inter-observer agreement of two radiologists was consistent with each other on *K* values, ranging from 0.71 to 0.95 for all images, and the excellent agreement between the two scoring radiologists was at 120 keV (*K* = 0.95).

**Figure 2:** The images of virtual monoenergetic images (VMI) and 120 kVp images. VMI of a 64-year-old male, from 50 keV to 140 keV. Approximately, 50–80 keV VMI displayed beam-hardening artifacts at the long-axis direction of nails. Approximately, 90–140 keV VMI showed that the artifacts became reduced gradually with the increase of keV and the brain structures near the nail became more visible. The 120 kVp images that displayed obviously beam-hardening artifacts at the level of stereotactic nails.

**Table 5:** Subjective image quality parameters.

**Energy level**	**Radiologist A**	**Radiologist B**	***Kappa*** **value**
120kVp	2.20 ± 0.48 (1–3)	2.18 ± 0.48 (1–3)	0.78
50keV	1.13 ± 0.35 (1–2)	1.17 ± 0.38 (1–2)	0.71
60keV	1.17 ± 0.38 (1–2)	1.17 ± 0.38 (1–2)	0.76
70keV	1.60 ± 0.56 (1–3)	1.60 ± 0.56 (1–3)	0.72
80keV	2.07 ± 0.58 (1–3)	2.10 ± 0.61 (1–3)	0.78
90keV	2.37 ± 0.56 (2–4)	2.40 ± 0.56 (2–4)	0.75
100keV	2.70 ± 0.65^a^(2–4)	2.73 ± 0.64^a^(2–4)	0.71
110keV	3.23 ± 0.63^a^(3–5)	3.83 ± 0.69^a^(3–5)	0.74
120keV	4.33 ± 0.48^a^(4–5)	4.40 ± 0.50^a^(4–5)	0.95
130keV	4.10 ± 0.55^a^(3–5)	4.20 ± 0.66^a^(3–5)	0.89
140keV	3.80 ± 0.66^a^(3–5)	3.93 ± 0.78^a^(3–5)	0.83

a *Represented that the subjective evaluation at this keV was statistically significant compared with 120 kVp images (p < 0.05)*.

## Discussion

In this study, the improvement on image quality and radiation exposure was analyzed between single- and dual-energy mode acquisitions to brain CT with stereotactic head frames using third-generation DSCT scanners. Our results verified that the dual-energy mode does not increase radiation exposure compared to the single-energy mode. Moreover, radiation dose reduction did not bring down the objective or subjective image quality based on our evaluation. Of note, we found that 120–140 keV VMI simultaneously decreased image noise by approximately 46–52% and increased SNR, CNR by approximately 139–196% and 98–110%. The subjective scores of 110–140 keV did reach a significant difference compared with that of 120 kVp images.

Metal artifacts reduction has long been a problem for radiologists and researchers since the birth of CT equipment. It is caused by the photon starvation effect and beam hardening effect. Some researchers have investigated direct in the ability to remove metal artifacts of dual-energy mode CT acquisitions with monochromatic imaging results (11–17). Magarelli et al. (18) performed the study that assessed image quality of dual-energy CT to reduce metal artifacts in subjects with knee and hip prostheses. The authors claimed that dual-energy CT with dedicated post-processing may reduce artifacts and significantly improve image quality. But comparison on the radiation exposure and image quality with a single-energy CT mode was missing in this study. Dong et al. (19) found image quality significantly increases to reduce artifacts for patients with the pedicle screws implants between the dual-energy mode (80/140 kVp) and the single-energy mode (140 kVp), and they pointed the optimal energy level was at 120 keV, which was consistent with our research, but they did not answer if the dual-energy mode had higher radiation exposure to get the better image quality. However, since the implementation of DSCT applications in clinical practice is growing, concerns about increased radiation dose delivered by two X-ray beam sources have been raised.

The two main concerns in this study were the image quality and radiation dose. The third-generation DSCT adds a tin filter placed in front of the X-ray tubes in order to absorb the low-energy photons and shift the polychromatic X-ray spectrum toward higher energy. These low-energy photons are usually responsible for the increase in image noise and the degradation of image quality (20). Also, it can cause unnecessary additional radiation to the patient. Another technical development for radiation reduction in DSCT is the using of the CARE Dose4D technique. CARE Dose4D is a four-dimensional automatic real-time dose adjustment technology, which can determine the size of patients according to the positioning image. X-ray tubes automatically output the required tube current value and CT dose index at low- and high-tube voltages so that the excellent image quality can be obtained at the lowest possible radiation dose when scanning different areas (21). Furthermore, it had been shown that high pitch can reduce radiation exposure without affecting image quality in previous studies (22, 23). In our study, the pitch of the dual-energy mode was higher than that of the single-energy mode. The combination of these techniques resulted in improved image quality and reduced radiation dose in the dual-energy mode.

In our results, the ED for the dual-energy mode was only (1.73 ± 0.45) mSv, nearly half the radiation dose of the single-energy mode. However, the images of the dual-energy mode better showed the structures in the brain. As shown in Table 4, CT values of the brain tissue near the steel nails were reduced due to the metal artifacts. The VMI did not work well at low energy level; low keV (50–80 keV) reconstruction also demonstrates the lower image quality compared to the single-energy images. But as the keV increased, it was above 110 keV images that were effective in removing metal artifacts. In terms of SNR, CNR, 110–40 keV VMI demonstrates a statistically significant advantage compared to 120 kVp images within the brain tissue. Unlike Selles M et al. (24) and Schmidt AMA et al. (25), we pointed that VMI at 120 keV was the optimal energy level, which could not only reduce obviously metal artifacts but also ensure image quality, which is an optimal monoenergetic image choice for DBS.

There are also a number of limitations in this study. First, the delineation of the ROIs is based on the observer's subjective judgment of the artifacts, so there is a potential selection bias. Second, both dual-energy and single-energy images were acquired from one scanning system (DSCT); therefore, no comparison was made between dual-energy and single-energy imaging algorithms in the SECT. Third, we have only evaluated 50–140 keV monoenergetic images; higher keV images have not been included, because the image quality is significantly degraded at 150–190 keV.

In conclusion, the results of our study suggested that the dual-energy mode monoenergetic images (120 keV) in brain CT of patients with stereotactic head frame provide overall excellent objective and subjective image quality at lower radiation dose compared to the single-energy mode.

## Data Availability Statement

The original contributions presented in the study are included in the article/supplementary material, further inquiries can be directed to the corresponding author.

## Ethics Statement

The studies involving human participants were reviewed and approved by Institutional Review Board of XuanWu Hospital of Capital Medical University. The patients/participants provided their written informed consent to participate in this study.

## Author Contributions

XZ designed the study and participated in methodology, formal analysis, investigation, and writing—original draft preparation. WC participated in methodology and formal analysis. JLi and CZ participated in formal analysis and investigation. MZ and YS participated in conceptualization, writing, review, and editing. JLu participated in conceptualization, writing, review, editing, and funding acquisition. All authors contributed to the article and approved the submitted version.

## Funding

This work was supported by the Beijing Municipal Administration of Hospitals, Ascent Plan [DFL20180802] and Beijing Natural Science Foundation [Z190014].

## Conflict of Interest

The authors declare that the research was conducted in the absence of any commercial or financial relationships that could be construed as a potential conflict of interest.

## Publisher's Note

All claims expressed in this article are solely those of the authors and do not necessarily represent those of their affiliated organizations, or those of the publisher, the editors and the reviewers. Any product that may be evaluated in this article, or claim that may be made by its manufacturer, is not guaranteed or endorsed by the publisher.

## References

[1] HeoYJKimSJKimHSChoiCGJungSCLeeJK. Three-dimensional fluid-attenuated inversion recovery sequence for visualisation of subthalamic nucleus for deep brain stimulation in Parkinson's disease. Neuroradiology. (2015) 57:929–35. 10.1007/s00234-015-1555-z26156865

[2] LiDZhangCGaultJWangWLiuJShaoM. Remotely programmed deep brain stimulation of the bilateral subthalamic nucleus for the treatment of primary parkinson disease: a randomized controlled trial investigating the safety and efficacy of a novel deep brain stimulation system. Stereotact Funct Neuro. (2017) 95:174–82. 10.1159/00047576528571034

[3] MetmanLVPalGSlavinK. Surgical treatment of parkinson's disease. Curr Treat Options Neurol. (2016) 18:49–64. 10.1007/s11940-016-0432-327739021

[4] KinfeThomas M. Stereotactic MR-guided focused ultrasound deep brain lesioning: the resurrection of posteroventral pallidotomy and thalamotomy for Parkinson's disease? Acta Neurochirurgica. (2017) 159:1367–69. 10.1007/s00701-017-3161-928364273

[5] BarnaureIPollakPMomjianSHorvathJLovblad KOBoëxC. Evaluation of electrode position in deep brain stimulation by image fusion (MRI and CT). Neuroradiology. (2015) 57:903–8. 10.1007/s00234-015-1547-z26022355

[6] NarutoNItohTNoguchiK. Dual energy computed tomography for the head. JJR. (2018) 36:69–80. 10.1007/s11604-017-0701-429119457

[7] CiceroGAscentiGAlbrechtMHBlandinoACavallaroMD'AngeloT. Extra-abdominal dual-energy CT applications: a comprehensive overview. Radiol med. (2020) 125:384–97. 10.1007/s11547-019-01126-531925704

[8] GinatDTMayichMDaftari-BesheliLGuptaR. Clinical applications of dual-energy CT in head and neck imaging. Eur Arch OtorhinolaryngoL. (2016) 273:547–53. 10.1007/s00405-014-3417-425472819

[9] Wouter vanEGuillaumeLMarcoDFrankV. Dual energy CT in radiotherapy:currentapplications and futureoutlook. Radiother Oncl. (2016) 119:137–44. 10.1016/j.radonc.2016.02.02626975241

[10] DeCCasselmanJVanHTDierensMVereeckeEBossuN. Analysis of metal artifact reduction tools for dental hardware in CT scans of the oral cavity: kVp, iterative reconstruction, dual-energy CT, metal artifact reduction software: does it make a difference. Neuroradiology. (2015)57:841–9. 10.1007/s00234-015-1537-125929982

[11] GuzińskiMWaszczukŁSasiadekMJ. Head CT. Image quality improvement of posterior fossa and radiation dose reduction with ASiR - comparative studies of CT head examinations. Eur Radiol. (2016) 26:3691–6. 10.1007/s00330-015-4183-426803506PMC5021717

[12] DunetVBernasconiMHajduSDMeuliRADanielRTZerlauthJB. Impact of metal artifact reduction software on image quality of gemstone spectral imaging dual-energy cerebral CT angiography after intracranial aneurysm clipping. Neuroradiology. (2017) 59:845–52. 10.1007/s00234-017-1871-628752310

[13] BoosJFangJHeidingerBHRaptopoulosVBrookOR. Dual energy CT angiography: pros and cons of dual-energy metal artifact reduction algorithm in patients after endovascular aortic repair. Abdom Radiol (NY). (2017) 42:749–58. 10.1007/s00261-016-0973-727896386

[14] WellenbergRHHDondersJCEKloenPBeenenLFMKleipoolRPMaasM. Exploring metal artifactreduction using dual-energy CT with pre-metal and post-metal implant cadaver comparison: are implant specific protocols needed. Skeletal Radiol. (2018) 47:839–45. 10.1007/s00256-017-2750-228842739PMC5915501

[15] KasparekMFTöpkerMLazarMWeberMKasparekMMangT. Dual-Energy CT and ceramic or titanium prostheses material reduce CT artifacts and provide superior image quality of total knee arthroplasty. Knee Surg Sports Traumatol Arthrosc. (2019) 27:1552–61. 10.1007/s00167-018-5001-829881885PMC6527539

[16] MeinelFGBischoffBZhangQWBambergFReiserMFJohnsonTRC. Metal artifact reduction by dual-energy computed tomography using energetic extrapolation: a systematically optimized protocol. Invest Radiol. (2019) 47:406–14. 10.1097/RLI.0b013e31824c86a322659595

[17] NairJRDeBloisFOngTDevicSTomicNBekeratH. Dual-energy ct: balance between iodine attenuation and artifact reduction for the evaluation of head and neck cancer. J Comput Assist Tomogr. (2017) 41:931–6. 10.1097/RCT.000000000000061728448423

[18] MagarelliNDeSVMarzialiGMenghiABurrofatoAPedoneL. Application and advantages of monoenergetic reconstruction images for the reduction of metallic artifacts using dual-energy CT in knee and hip prostheses. Radiol Med. (2018) 123:1–8. 10.1007/s11547-018-0881-829637389

[19] DongYShiAJWuJLWangRXSunLFLiuAL. Metal artifact reduction using virtual monoenergetic images for patients with pedicle screws implants on CT. Eur Spine J. (2016) 25:1754–63. 10.1007/s00586-015-4053-426070548

[20] LengaLTrappFAlbrechtMHWichmannJLJohnsonAAYelI. Single- and dual-energy ct pulmonary angiography using second- and third-generation dual-source ct systems: comparison of radiation dose and image quality. Eur Radiol. (2019 29:4603–612. 10.1007/s00330-018-5982-130666446

[21] WangLGongSYangJZhouJXiaoJGuJH. Care dose 4d combined with sinogram ffirmed iterative reconstruction improved the image quality and reduced the radiation dose in low dose ct of the small intestine. J Appl Clin Med Phy. (2018) 20:293–307. 3050827510.1002/acm2.12502PMC6333130

[22] ApfaltrerGAlbrechtMHSchoepfUJDuguayTMDe CeccoCNNanceJW. High-pitch low-voltage CT coronary artery calcium scoring with tin filtration: accuracy and radiation dose reduction. Eur Radiol. (2018) 28:3097–104. 10.1007/s00330-017-5249-229404770

[23] SuntharalingamCMikatAWetterNGuberinaASalem P HeilP. Whole-body ultra-low dose CT using spectral shaping for detection of osteolytic lesion in multiple myeloma. Eur Radiol. (2018) 28:2273–80. 10.1007/s00330-017-5243-829322333

[24] SellesMStuivenbergVHWellenbergRHHvan de RietLNijholtIMvan OschJAC. Quantitative analysis of metal artifact reduction in total hip arthroplasty using virtual monochromatic imaging and orthopedic metal artifact reduction, a phantom study. Insights Imaging. (2021) 12:171. 10.1186/s13244-021-01111-534817722PMC8613319

[25] SchmidtAMAGrunzJPPetritschBGruschwitzPKnarrJHuflageH. Combination of iterative metal artifact reduction and virtual monoenergetic reconstruction using split-filter dual-energy CT in patients with dental artifact on head and neck CT. AJR Am J Roentgenol. (2022) 218:716–727. 10.2214/AJR.21.2677234755521

